# Application of Computer 3D Modeling Technology in Graphic Image Design

This article has been retracted.

**DOI:** 10.1155/2022/6451339

**Published:** 2022-07-16

**Authors:** Jin Liu

**Affiliations:** Department of Animation and Art, Zibo Vocational Institute, Zibo 255000, Shandong, China

## Abstract

In order to solve the problem that the manual input data work efficiency is low and the optimization cannot be achieved in the section modulus calculation, the author proposes a computer-aided 3D graphic design method for ship hull structure. First, complete the modeling of the ship hull, complete the statistical calculation of the size in the CAD platform, solve the static moment, and complete the three-dimensional modeling; Calculate the inertial load and wave load of the ship during work, and calculate the wave bending moment, and substitute it into the three-dimensional model for verification. Finally, according to the computer-aided three-dimensional graphic design process, the specification verification of the ship's scale is completed, the graphic file is associated with the database, and the three-dimensional graphic design is completed. Experimental results show that the maximum stress of the original three-dimensional integrated graphic design of the ship is 202 MPa, and the maximum deformation is 87.352 mm. Based on the computer-aided three-dimensional integrated graphic design of the ship, the maximum stress is 226 MPa, and the maximum deformation is 76.234 mm. *In conclusion*: the hull obtained by the computer-aided three-dimensional graphic design of the ship can effectively reduce the total area and materials of the midsection structure of the ship, reduce the weight of the hull, and realize the optimal configuration of the midsection material of the ship.

## 1. Introduction

Shipbuilding is a modern comprehensive industry that provides technical equipment for water transportation, marine development, and national defense construction. It is a strategic industry combining military and civilians, and an important part of advanced equipment manufacturing, further strengthening of the shipbuilding industry is an inevitable requirement to improve China's comprehensive national strength. He is of great significance to safeguarding national maritime rights and interests, accelerating maritime development, ensuring strategic transportation safety, promoting sustained national economic growth, and increasing employment [1]. Judging from the changes in the share of China's shipbuilding industry in the world shipbuilding market in the past ten years, the share of China's shipbuilding industry in the global market is rising sharply, and China has become one of the world's important shipbuilding countries. The industrial transfer trend of international manufacturing is the biggest opportunity for the development of China's shipbuilding industry. However, affected by the deep adjustment of the international shipping market, deep-seated problems such as “difficulty in financing”, “difficulty in delivery” and “difficulty in making profits” still exist, and the shipbuilding industry is still facing a severe situation [2]. Therefore, in the fierce market competition environment, how to avoid various risks and how to seize opportunities are very important to the development of enterprises.

Since 2010, China has ranked first in the world in terms of shipbuilding completions, new orders, and orders in hand for three consecutive years. However, we must be soberly aware that although China's shipbuilding industry is developing rapidly, many contradictions and problems have also accumulated. Compared with advanced shipbuilding countries such as Japan and South Korea, its main features are a long shipbuilding cycle, weak innovation ability, prominent structural contradictions, and low industrial concentration, the production efficiency and management level need to be improved, the development of the ship supporting industry is lagging behind, the development of marine engineering equipment is slow, the design and development capability is insufficient, the ship type development capability is weak, and the precision control technology is weak [3]. The long shipbuilding cycle is one of the important factors restricting the rapid development of China's shipbuilding industry, and the quality of the design and the length of the cycle are also important factors that determine the length of the shipbuilding cycle. How to effectively shorten the cycle and improve the quality in the ship design stage has become the focus of research.

## 2. Literature Review

Computer-aided design technology can improve the efficiency and quality of ship design, which has been recognized by the domestic shipbuilding industry. Some international advanced 3D shipbuilding software has also been introduced in China, and at the same time, there are also researchers who have carried out secondary development of the corresponding 3D software, and an easy-to-use ship digital design platform is designed [4]. The digitization of the ship design process is to use technologies such as virtual design to realize the digitization of product design methods and design processes, shorten the product development cycle, and improve the product innovation capability of enterprises. Bagz et al. studied through the secondary development technology to achieve three-dimensional, in the design of the main hull, the ship wall, cabin modeling, structural modeling, and ship capacity calculation functions [5]. Li et al. used secondary development technology and curve surface technology to study the application technology of 3D modeling of ships [6]. Petacco et al., relying on workstations and graphic support software, completed the definition and design process of specific models in ship-aided design, verifying that virtual assembly technology can effectively shorten the production design cycle of ships [7]. Meshalkin et al. used the sample design method to select the appropriate reference mother ship and transformed the designer's experience and heuristic knowledge into a readable format, which was integrated into the computer system software for the ship concept design stage [8]. Lee et al. reviewed the research of expert system in ship design and manufacture, and it is pointed out that the ship design and manufacturing industry need the expert system to improve the efficiency [9]. Hao et al. applied the system-based intelligent design method to the ship's engine and ship layout, designed and developed a system, pointed out that the design efficiency of the original computer-aided design system can be significantly improved in the preliminary design stage and the overall design stage of the ship, and further expanded the functions of the existing system [10].

In order to enhance the competitiveness of my country's ships in the international market, while improving the quality of ships, we must also consider the design accuracy and design cycle, my country's large and medium-sized shipbuilding enterprises have introduced 3D shipbuilding software, but this software cannot be applied to domestic processes, and the accuracy and work efficiency of traditional design methods have been severely challenged. In the early stage of ship design, the section modulus calculation and other structural design calculation are needed. Although some AIDS are used, they are only semiautomated tools. There is a need to manually input the data which restricts the efficiency of the work, resulting in the middle section material configuration not optimal. So, this paper designs a 3D graphic design method of the ship hull structure based on computer-aided design technology.

## 3. Research Methods

### 3.1. Generate Component Library

3D modeling is the basis of 3D printing; that is, the product needs to be modeled in 3D software before printing, so 3D printing requires the participation of computer-aided design (CAD) technology. The conceptual design of the database refers to the concept class in the domain model in the demand analysis stage or the related objects in the real world, the process of abstracting and expressing with the help of a certain database conceptual model. The conceptual design is independent of the type and details of the database and is an intermediary between the real world and the information world. It can fully express and reflect the entities in the real world and the relationship between entities, and at the same time, it can convert to the logical model of various databases. Therefore, the conceptual structure of the database is easy to understand, and it is convenient for developers to exchange opinions with users who are not familiar with computers, so that the design process of the database is closer to the needs of users.

In order to make up for the deficiencies of traditional databases in dealing with complex objects, engineering databases complement traditional hierarchical, mesh, and relational data models, in order to meet the requirements of expressing the full semantic structure of engineering data [11]. The engineering data model can be divided into expanding the traditional database model, including expanding the mesh data model, expanding the relational data model (such as XSQL and NF2 expanding the relational data model), and the object-relational model; special engineering data models such as function data model, version model, and semantic data model include general object-oriented model and special semantic data model (such as statistics-oriented SAM*∗* model and CAD/CAM integration-oriented object model) [12].

First, the component library of the ship structure is constructed, including the end cutting library, opening library, bracket library, profile library, and plate library. Its overall structure is shown in Figure 1.

Add construction parameter information to the graphic 3D information base and realize the construction of three-dimensional integrated graphics component library for ships [13]. The component parameters of the component library are shown in Table 1.

### 3.2. Ship Hull Modeling

Digital modeling is not the same as manual modeling using software. Using software to manually model, it is easy to control every detail of the model, but its disadvantage is that it takes too long; especially in engineering applications, if you want to get a 3D model of the product, you need the help of digital modeling. The realization of digital modeling is that programmers compile the design work into easy-to-operate software using various secondary development languages according to the needs of the project [14]. Using this software, you can quickly get a design model with simple data input, without knowing how to extrude, trim surfaces, etc. The establishment of the three-dimensional model of the hull can accurately and effectively solve the corresponding loads of the hull components and complete the overall strength calculation of the ship. The range of models used by different ship classes has different requirements.

As can be seen, the section is composed of multiple components, BL is the baseline, and it is used as the coordinate axis *x*, which is positive to the head, and the center line CL is the *y*-axis, which is positive from the longitudinal section to the left. The development platform chooses CAD, and after the CAD construction is selected, it is necessary to carry out relevant dimension calculation and statistics [15]. The cross-sectional area of a certain member is when the cross-sectional area and centroid coordinates are known, the static moments of the cross section with respect to the *y*-axis and the *x*-axis can be obtained as follows:

(1) $$\begin{array}{c} \left\{\begin{array}{c} S_{y}=Ax_{c},\\ S_{x}=Ay_{c}. \end{array}\right. \end{array}$$

In the formula, *x*_*c*_ and *y*_*c*_ are the centroid coordinates of the section, and the static moment of the section to a certain axis can be expressed as the sum of the static moments of the components of the section relative to the coordinate axis. Therefore, the static moment of the entire section can be expressed as the following formula:

(2) $$\begin{array}{c} \left\{\begin{array}{c} S_{y}=\sum A_{i}x_{ci},\\ S_{x}=\sum A_{i}y_{ci}, \end{array}\right. \end{array}$$

where *A*_*i*_, *x*_*ci*_, *y*_*ci*_ represent the area and centroid coordinates of each component in the section, respectively. Based on the above calculations, a three-dimensional model of the ship's hull structure can be constructed.

The obtained 3D model not only establishes the three-dimensional model of the ship but also includes various production and process information, such as shrinkage allowance, welds, and grooves, and this additional information lays the foundation for the later production of the hull [16].

### 3.3. Calculated Loads

During the process of loading and sailing at sea, the ship will be subjected to the force of multiple loads, and it mainly includes cargo load, corresponding inertial load, and sea wave load. The accuracy of the calculation of these loads determines the accuracy of the ship's structural strength assessment [17]. When a ship sails on water, it will be subjected to still water loads and wave loads. The weight including the hull is decomposed along a certain direction, divided into trapezoidal weight distribution, and superimposed one by one to form a weight distribution curve. The additional bending moment of the middle arch wave can be calculated as the following formula:

(3) $$\begin{array}{c} M_{WH}=0.5h\cdot K_{B}\cdot A_{1}\cdot A_{2}\cdot BL^{2}\times 10^{-2},\\ K_{B}=\left(0.56+0.4\alpha \right)\left[0.025+0.032\left(\frac{C_{b}}{\alpha }\right)-0.6\right], \end{array}$$

where *h* is the wave height, *K*_*B*_ is the coefficient considering the influence of the line shape, *A*_1_ is the influence coefficient considering the actual still water bending moment of the ship sailing, *A*_2_ is the hydrodynamic pressure correction coefficient, B is the waterline width at midship at normal displacement, and *L* is the design waterline length. The formula for calculating the additional bending moment of midsag waves is as follows:

(4) $$\begin{array}{c} M_{WS}=0.5h\cdot K_{B}\cdot A_{1}\cdot A_{2}\cdot BL^{2}\times 10^{-2},\\ K_{B}=1.437\alpha \left[0.032+0.013\left(\frac{C_{b}}{\alpha }\right)-0.6\right], \end{array}$$

where *C*_*b*_ represents the square coefficient, and the calculation formula of the vertical slamming moment can be expressed as the following formula:

(5) $$\begin{array}{c} M_{DS}=0.5h\cdot K\cdot B^{2}L\times 10^{-2},\\ K=0.1338\sqrt{\frac{L}{T}}-0.4486. \end{array}$$

The other parameters in the formula are the same as the calculation of the additional bending moment of the middle arch, and the calculation formula of the slamming moment of the middle arch can be expressed as the following formula:

(6) $$\begin{array}{c} M_{DH}=0.4M_{DS}. \end{array}$$

The values calculated above can be substituted into the established ship model for verification.

### 3.4. 3D Structural Design of Ships

After the component library is generated, the three-dimensional structure of the ship is designed using computer-aided functions. Include importing hull surfaces, deck generation, stiffener arrangements, and openings. To input the hull surface, it is necessary to obtain the relevant information such as the ship hull size, perform diffraction transformation on the size data to generate the hull surface, and input it into the computer-aided system [18].

The generation of the deck needs to determine the deck parameters such as thickness, start and end rib, and height. It is also necessary to select the type and material of the deck in the plate library. Deck parameters are defined by CATIA, and the deck model is semantically marked by EKL language. Among them, the thickness and material of the board should be selected. After the deck is generated, the rule base will automatically name the generated ship deck through the naming rules.

The arrangement of the reinforcing ribs needs to select the type to which they belong, set the positioning method, welding line, and the specific model of the profile, and call the profile library [19]. The orientation and position of the profiles are adjusted according to the positioning parameters, and the material properties and arrangement of the reinforcing ribs are set to complete the arrangement. When the reinforcement rib passes through the bulkhead, it must be punched. The shape of the perforation is determined by the specific type of bulkhead and the cross-sectional shape of the stiffener. Therefore, it is necessary to match the opening library, plate library, and section library. When matching, it is necessary to define a rule base and set the associated parameters [20].

### 3.5. Computer-Aided Three-Dimensional Graphic Design of Ship Structure

After the above calculation is completed, input the length data of the ship's hull, and the horizontal distance from the bilge to the intersection of the midlongitudinal section and 10 stations, and according to the design specification of the ship, the scale specification of the ship is verified according to the corresponding process, and the process is shown in Figure 2.

The designed graphic file is associated with the database. After using the section modulus calculation program to create a new calculation project, it is necessary to specify the associated CAD graphics file for the project, so that the designer can specify the primitives to be calculated in CAD and record the information, and complete the operations such as opening and drawing related to 3D graphics.

### 3.6. Experiment

In order to verify the validity of the three-dimensional graphic design method of the ship hull structure designed by the author, an actual ship calculation example is required. The 3D graphic design method studied in this paper is used to optimize the midsection structure of a certain ship. Using computer-aided three-dimensional integrated graphics of ships, and the original three-dimensional integrated graphics design method of ships, the three-dimensional integrated graphics of ships and ships are designed separately. Analyze the performance of the two design methods for manufacturing, obtain the maximum stress and maximum deformation data of the designed ship, and compare the effects of the three-dimensional integrated graphics of the ship. The judgment is based on the maximum stress and maximum deformation of the designed ship graphics. Among them, the larger the stress and the smaller the deformation, the better the effect of the three-dimensional integrated graphic design of the ship. On the contrary, the smaller the stress and the greater the deformation of the three-dimensional integrated graphic design of the ship, the less effective the three-dimensional integrated graphic design of the ship is [21].

The relevant parameters of the hull are as follows: the maximum length of the hull is 154 m, the design waterline width is 16.3 m, the length between the vertical lines is 140 m, the design draft is 4.72 m, the maximum width of the fold line is 17.1 m, the maximum deck width is 16.8 m, and the molding depth and beam arch are 10.3 m and 0.168 m, respectively.The hull material is steel, with a density of 7 800 kg/m3, a Young's modulus of 2.10 ell Pa, and a Poisson's ratio of 0.3. According to the force analysis of each part of the ship structure, in the experiment, the midship section can be refined and classified, and it is mainly divided into the side shell, each deck, the inner bottom, and the outer bottom, and the author directly selects the actual proportional relationship of the above-mentioned ships to conduct experiments [22].

## 4. Analysis of Results

For the convenience of comparison, in the experimental results, the original design value and the author's design value are counted and compared, as shown in Figure 3.

As can be seen, using the three-dimensional graphic design method studied by the author, the first-level optimization of the midsection of the ship can be realized, and the designed hull can effectively reduce the total area and materials of the midship section structure, reduce the weight of the hull, and realize the optimal configuration of the midsection material of the ship, which shows that the author's method has certain effectiveness.

Table 2 shows the effect of the original three-dimensional integrated graphic design of the ship.

Table 3 shows the design effect of the computer-aided three-dimensional integrated graphics of the ship.

By comparison, it can be seen that the maximum stress of the original three-dimensional integrated graphic design of the ship is 202 MPa, and the maximum deformation is 87.352 mm. Based on the computer-aided three-dimensional integrated graphic design of the ship, the maximum stress is 226 MPa, and the maximum deformation is 76.234 mm. By comparing the data, it can be seen that the effect of the computer-aided three-dimensional integrated graphics of the ship is superior to the original three-dimensional integrated graphic design method of ships, which verifies the effectiveness of the author's method [23].

## 5. Conclusion

The configuration optimization of the material in the middle section of the ship is mainly based on the CAD interactive calculation program, which changes the shortcomings of the previous semiautomatic manual data input, improves the work efficiency and the calculation efficiency of the graphic design, and effectively completes the graphic design optimization of the middle section in the three-dimensional graphic design of the ship, effectively reducing the hull cabin material and weight and save cost. However, the author's structural optimization module only supports grain and modal analysis, so only the strength check is carried out in the process of graphic design, and the check analysis of buckling and other aspects is also lacking. This problem needs to be solved in future research.

## Figures and Tables

**Figure 1:** Composition of the build library.

**Figure 2:** The process of computer-aided 3D graphic design.

**Figure 3:** Comparison of design variables.

**Table 1:** Component parameters of component library.

name	Targeting parameters	Shape parameters	Simplified features	Attributes	Category affiliation
Plate library	Upper and lower	Thickness	First/second order	Material	Deck/Shell/Bulkhead
Profile library	Right beam, left beam	Net, rim	Standard section	Material	Panel
Toggle library	Right beam, left beam	Hole, thickness	Plate	Material	Rod, panel
Opening library	Centroid	Length	Washer	-	Panel
End cutting library	-	Length, angle	Standard section	Material	Panel

**Table 2:** Experimental results of the original three-dimensional integrated graphics of ships.

	Maximum stress/MPa	Max deformation/mm
Allowance	284	132
Calculated	202	87.352
Safety	Safety	Safety

**Table 3:** The experimental results of the three-dimensional integrated graphics of the ship designed by the author.

	Maximum stress/MPa	Max deformation/mm
Allowance	284	132
Calculated	226	76.234
Safety	Safety	Safety

## Data Availability

The data used to support the findings of this study are available from the corresponding author upon request.
